This article has been retracted.

# Coding and Noncoding RNA Expression Profiles of Spleen CD4^+^ T Lymphocytes in Mice with Echinococcosis

**DOI:** 10.1155/2022/9742461

**Published:** 2022-04-08

**Authors:** Songhao Yang, Xiancai Du, Chan Wang, Tingrui Zhang, Shimei Xu, Yazhou Zhu, Yongxue Lv, Yinqi Zhao, Mingxing Zhu, Lingna Guo, Wei Zhao

**Affiliations:** ^1^Key Laboratory of Prevention and Control of Common Infectious Diseases of Ningxia Hui Autonomous Region, Ningxia Hui Autonomous Region 750004, Yinchuan, China; ^2^Department of Medical Genetics and Cell Biology, School of Basic Medical Science of Ningxia Medical University, Ningxia Hui Autonomous Region 750004, Yinchuan, China; ^3^Center of Scientific Technology of Ningxia Medical University, Ningxia Hui Autonomous Region 750004, Yinchuan, China

## Abstract

Cystic echinococcosis (CE) is a severe and neglected zoonotic disease that poses health and socioeconomic hazards. So far, the prevention and treatment of CE are far from meeting people's ideal expectations. Therefore, to gain insight into the prevention and diagnosis of CE, we explored the changes in RNA molecules and the biological processes and pathways involved in these RNA molecules as *E. granulosus* infects the host. Interferon (IFN)-*γ*, interleukin (IL)-2, IL-4, IL-6, IL-10, IL-17A, and tumor necrosis factor (TNF)-*α* levels in peripheral blood serum of *E. granulosus* infected and uninfected female BALB/*c* mice were measured using the cytometric bead array mouse Th1/Th2/Th17 cytokine kit. mRNA, microRNA (miRNA), long noncoding RNA (lncRNA), and circular RNA (circRNA) profiles of spleen CD4^+^ T cells from the two groups of mice were analyzed using high-throughput sequencing and bioinformatics. The levels of IFN-*γ*, IL-2, IL-4, IL-6, IL-10, IL-17A, and TNF-*α* were significantly higher in the serum of the CE mice than in control mice (*P* < 0.01). In total, 1,758 known mRNAs, 37 miRNAs, 175 lncRNAs, and 22 circRNAs were differentially expressed between infected and uninfected mice (|fold change| ≥ 0.585, *P* < 0.05). These differentially expressed molecules are involved in chromosome composition, DNA/RNA metabolism, and gene expression in cell composition, biological function, and cell function. Moreover, closely related to the JAK/STAT signaling pathways, mitogen-activated protein kinase signaling pathways, P53 signaling pathways, PI3K/AKT signaling pathways, cell cycle, and metabolic pathways. *E. granulosus* infection significantly increased the levels of IFN-*γ*, IL-2, IL-4, IL-6, IL-10, IL-17A, and TNF-*α* in mouse peripheral blood of mice and significantly changed expression levels of various coding and noncoding RNAs. Further study of these trends and pathways may help clarify the pathogenesis of CE and provide new insights into the prevention and treatment of this disease.

## 1. Introduction

Cystic echinococcosis (CE) refers to a serious zoonotic parasitic disease caused by *Echinococcus granulosus* [1, 2]. Dogs are the final host and the main source of infection. Direct infection is due to the close contact between people and dogs, and the oral infection occurs after the insect eggs on their fur pollute their fingers. In animal husbandry areas, sheep are the main intermediate host. The insect eggs in dog feces pollute the pasture, infect the sheep, and complete the life cycle among livestock. People do not infect each other, and the intermediate host will not infect the intermediate host. The prevalence of echinococcosis among intermediate hosts has caused huge economic losses to the production and development of local animal husbandry. The high incidence areas of CE are mainly concentrated in western China (Tibet, Qinghai, Gansu, and Ningxia), southern America, and East Africa [3, 4]. The target organs of CE are mainly the liver and lungs but also the brain, spleen, kidneys, heart, and spine. Notoriously, CE cysts develop very slowly, and the disease may be asymptomatic for 10–15 years [5, 6]. As a result, patients with CE often present to the hospital late, which prevents early disease management. There have been significant advances in the study of CE in recent years; however, imaging is still the main diagnostic tool, and it is difficult to identify cysts of less than 2 cm in diameter [7–9]. Clinically, serum testing can support the diagnosis of CE, but unfortunately, the sensitivity and specificity of the tests are low, and there are major limitations in terms of the prognosis [10, 11]. Data on the underlying mechanisms involved in the development and progression of CE in the host are scarce. Thus, given the limitations of the current diagnostic techniques, the ineffectiveness of drugs, and the inadequacy of surgery, there is an urgent need to explore molecular mechanisms and related pathways involved in the progression of CE to identify new drug and vaccine targets.

RNA is a macromolecule that plays an important biological role in the coding, decoding, regulation, and expression of genes [12]. Based on various functions, RNA can be divided into coding and noncoding RNA (ncRNA). In particular, mRNA is a transmitter of genetic information that directs protein synthesis. RNAs that cannot have the ability to encode proteins (ncRNAs) can be classified according to their length into miRNAs (18–24 nucleotides) and long ncRNAs (lncRNAs), which similar to circular RNAs (circRNAs), are >200 nucleotides in length [13, 14]. Recent studies have reported an increasing number of coding and ncRNAs that are widely expressed during tapeworms infection in hosts [15–18]. M. E Ancarola et al. reported for the first time that miRNAs can be secreted in the bladder of two tapeworms, which provides valuable data for the basic biological research of noncoding RNA of tapeworms [15]. Yu et al. found that there were dysregulated lncRNAs in the M-MDSCs of *E. granulosus* infection mouse models, they might be involved in M-MDSC-derived immunosuppression in related diseases [16]. These molecules may be key regulators of worm–host interactions. A search for potentially effective molecules and related pathways is expected to provide novel perspectives and a meaningful clinical value for diagnosing and treating helminthiasis.

Therefore, this study first prepared the mouse model of *E. granulosus* infection, then screened the differentially expressed coding and noncoding RNA molecules between infected mice and control mice by high-throughput sequencing and analyzed the biological processes and pathways involved in the differentially expressed coding and noncoding RNA molecules by bioinformatics, hoping to provide a basis for the basic research and clinical prevention and treatment of CE.

## 2. Materials and Methods

### 2.1. Parasite Infection

Protoscoleces of *E. granulosus* were obtained by surgical removal of cysts from patients with CE at the General Hospital of Ningxia Medical University, Department of Hepatobiliary Surgery. Twenty 6-week-old female BALB/*c* mice were purchased from the Ningxia Medical University Laboratory Animal Centre. The mice were randomly divided into two groups; mice in the infected group (*n* = 6) were intraperitoneally injected with 2,000 *E. granulosus* protoscoleces in phosphate-buffered saline (PBS) and mice in the uninfected group (*n* = 6) were intraperitoneally injected with an equal volume of PBS.

### 2.2. Cytokine Measurement in the Serum

Peripheral blood serum from two groups of mice (*n* = 10) was used to measure the levels of interferon (IFN)-*γ*, interleukin (IL)-2, IL-4, IL-6, IL-10, IL-17A, and tumor necrosis factor (TNF)-*α* using the cytometric bead array mouse Th1/Th2/Th17 cytokine kit (Becton, Dickinson and Company). The captured microspheres were mixed and centrifuged at 200 × g at room temperature for 5 min. The supernatant was aspirated, and an equal volume of a serum enhancement solution was added, followed by vortexing and incubation for 30 min at room temperature, protected from light. Subsequently, the mixture was added to an equal volume of serum, and all the tubes were incubated for 3 h at room temperature, protected from light, with equal amounts of a phycoerythrin-labeled antibody for cytokine detection.

### 2.3. Sample Isolation

Spleen CD4^+^ T cells from the infected and uninfected mice were isolated 6 months after infection by a mouse Splenic Lymphocyte Isolation Kit (TIAN JIN HAO YANG, LTS1092PK) and CD4^+^*T* Cell Isolation Kit (Miltenyi, 130-104-453). Total RNA was extracted from CD4+ T cells using the TRIzol reagent (Invitrogen) according to the manufacturer's instructions. RNA quality and purity were evaluated using a NanoDrop 2000c instrument (Thermo Fisher Scientific). The RevertAid first-strand cDNA synthesis kit (Thermo Fisher Scientific) was used for cDNA synthesis following the manufacturer's directions.

### 2.4. Coding and ncRNA Expression Profiles and Pathway Analysis

High-throughput RNA sequencing was performed by Shanghai Novelbio (China). The original data were manipulated to obtain high-quality reads. The RNA tags were exactly matched to the mouse genome to identify the known RNAs. The relative RNA expression levels in the two groups of mice were determined using the DESeq *R* package. The |fold change| ≥ 0.585 and *P* < 0.05 were used to identify differentially expressed RNAs. Volcano plots and heatmaps were used to visualize the differential RNA expression profiles between the two groups.

### 2.5. Statistical Analysis

All data were processed using GraphPad Prism 5 (GraphPad Software, La Jolla, CA, USA), and the *t*-test was used for comparison between the two groups of mice. Fisher's test was used to calculate the significance level of each Gene Ontology (GO) term to determine differentially significant GO terms and pathways. Statistical significance was set at *P* < 0.05.

## 3. Results

### 3.1. Serum Cytokine Levels in CE Mice

The levels of IFN-*γ*, IL-2, IL-4, IL-6, IL-10, IL-17A, and TNF-*α* were measured in the peripheral blood serum of 6 CE mice and 6 control mice and were found to be significantly higher in the CE mice than in the control group, as shown in Figure 1 (*P* < 0.01). IFN- *γ*, IL-2, and TNF- *α* participate in Th1-mediated cellular immune response; IL-4 and IL-6 participate in Th2-mediated humoral immune response; IL-17A participate in Th17-mediated immune response; Th1 and Th17 have a synergistic effect, and IL-10 participate in immune regulation. The immune response to *E. granulosus* is regulated by cellular immunity and humoral immunity. These findings suggest a strong immune response in mice to reject the parasitism of *E. granulosus*, even at 6 months after the infection. This shows that the mouse model of *E. granulosus* infection is successful, which enables further experiments.

### 3.2. Identification of Differentially Expressed Coding and ncRNAs in Association with *E. granulosus* Infection

To identify coding and ncRNAs associated with CE, spleen CD4^+^ T cells were isolated from two infected and two control mice 6 months post-infection. There were a total of 1,758 known differentially expressed mRNAs, 37 differentially expressed miRNAs, 175 differentially expressed lncRNAs, and 22 differentially expressed circRNAs between the two groups (|fold change| ≥ 0.585, *P* < 0.05), which are shown in the volcano and cluster plots.  Figure 2(a) and Figure 2(b) are volcano and cluster plots of mRNAs, respectively.  Figure 2(c) and Figure 2(d) are volcano and cluster plots of miRNAs, respectively.  Figure 2(e) and Figure 2(f) are volcano and cluster plots of lncRNAs, respectively.  Figure 2(g) and Figure 2(h) are volcano and cluster plots of circRNAs, respectively. The detailed information for the top 20 differentially expressed molecules of each type is presented in Tables.  Table 1 gives details of the first 20 differentially expressed mRNA molecules.  Table 2 shows the details of differentially expressed miRNAs molecules.  Table 3 shows the details of differentially expressed lncRNAs molecules.  Table 4 shows the details of differentially expressed circRNAs molecules. The expression of these molecules was significantly altered in the CE mice compared with that in the control mice, which suggested that these RNAs might be involved in the development of this parasitic disease.

### 3.3. GO and Pathway Analyses of Differentially Expressed Genes between CE and Normal Mice

The results of the high-throughput sequencing of the differentially expressed genes are further analyzed based on GO annotations to predict the biological processes, molecular functions, and cellular components that transcripts may participate in. The differentially expressed mRNAs between the CE mice and the control mice are mainly involved in the DNA replication-dependent nucleosome assembly, cell cycle, negative regulation of megakaryocyte differentiation, regulation of gene silencing, innate immune response in the mucosa, and immune system process in biological process as shown in Figure 3(a). It is important to participate in the protein heterodimerization activity, DNA binding, antioxidant activity, MHC class I protein complex binding, and ammonium transmembrane transporter activity in molecular function, as shown in Figure 3(a). In terms of cellular components, it is mainly involved in chromosome, nucleosome, kinetochore, cytoskeleton, and chromosome passenger complex as shown in Figure 3(a). Notably, these differentially expressed molecules are closely related to the glutathione metabolism, glycolysis/gluconeogenesis, glycerolipid metabolism, cell cycle, and the p53 signaling pathway as shown in Figure 3(b).

Results similar to mRNA showed that the circRNAs identified are primarily associated with the T-helper 1 cell lineage commitment, interleukin-4-mediated signaling pathway, positive regulation of isotype switching to IgE isotypes, miRNA catabolic process, and negative regulation of type 2 immune response in biological process as shown in Figure 3(c). It is important to participate in the nucleotidyltransferase activity, phosphatase regulator activity, tRNA guanylyltransferase activity, DNA primase activity, and DNA/RNA helicase activity in molecular function as shown in Figure 3(c). In terms of cellular components, it is mainly involved in spindle pole, kinetochore, PTW/PP1 phosphatase complex, spindle microtubule, and peroxisomal membrane as shown in Figure 3(c). Furthermore, the differentially expressed circRNAs are involved in the leukocyte transendothelial migration, Hippo, JAK/STAT, oxytocin, and cGMP/PKG signaling pathways as shown in Figure 3(d). These results suggest that these pathways might be promising targets for the treatment of CE.

### 3.4. Gene Act Network of Differentially Expressed mRNAs

Although we obtained important signaling pathways associated with CE, one gene could simultaneously be involved in multiple signaling pathways. Therefore, we constructed a gene act network based on the correlation between differentially expressed mRNAs, including their expression, binding, repression, activation, and complexes. This analytical approach can form corresponding regulatory affiliations, making it easier to identify important related genes. Analysis of the gene act network shows that all differentially expressed molecules between infected and uninfected mice were closely associated with the JAK/STAT, mitogen-activated protein kinase (MAPK), P53, and PI3K/AKT signaling pathways, cell cycle, and metabolic pathways as shown in Figure 4. In particular, three pathways, namely, the JAK/STAT, MAPK, and P53 signaling pathways, showed the largest numbers of arrows and maybe the most likely new targets for the treatment of CE.

## 4. Analysis and Discussion of Clinical Data

As a parasitic zoonosis, CE is prevalent in areas with well-developed livestock industries, especially sheep, and greatly hinders livestock productivity development and damages the regional economy [8]. Although albendazole has been used in the treatment of CE in recent decades, its efficacy has not been adequately demonstrated. Long-term use of benzimidazoles may cause a variety of adverse effects, especially in the liver [19–22], and the development of new alternative drugs would be of great importance for the treatment of CE. Following infection, echinococcosis activates a strong immune response in the host, eliminating most of the parasite within a few days [23]. Based on this, we constructed a mouse model of *E. granulosus* protoscoleces infection and detected differentially expressed mRNAs, lncRNAs, miRNAs, and circRNAs.

The progress in the study of differential expression profiles of RNA in both CE itself and in the infected host has been very limited in terms of molecular mechanisms. In vitro cultured *E. granulosus* protoscoleces, a total of 172 genes and 15 miRNAs, which are mainly involved in neurological development and carbohydrate metabolic processes, were shown to be significantly altered during development. In addition, miR-71 and miR-219 regulated genes may be involved in redox processes during adult development [24]. Whole-genome sequencing of *E. granulosus* identified 42 mature miRNAs in three different model stages [25]. It has been suggested that some molecules, such as miR-19b, miR-71, and miR-222-3p, could serve as possible biomarkers for *E. granulosus* [26, 27]. In hosts infected with *E. granulosus*, restimulation of the patient's peripheral blood mononuclear cells using crude *E. granulosus* antigens induced the expression of Th1/Th2 cytokine mRNAs [28, 29]. Differentially expressed miRNAs (miR-181, miR-30, miR-365, miR-378, miR-449, and miR-16) that were identified in the sheep intestine, liver, and serum, as well as in mouse macrophages, following infection with *E. granulosus* may be critically involved in the body's immune response [30–32]. Microarray analysis of circRNA expression profiles in adjacent tissues of CE-infected patients showed that hsa_circRNA_006773, hsa_circRNA_049637, hsa_circRNA_104349, and hsa_circRNA_406281 might serve as CE prognostic biomarkers and therapeutic targets [33]. Interestingly, lncRNA regulates lipolysis and metabolic remodeling in *E. granulosus*–infected mice [34]. Aberrant lncRNAs were found in myeloid-derived suppressor cells of infected mice, which may be associated with immunosuppression [16]. Microarray sequencing of exosome-like vesicles in human liver hydatid cysts revealed that miRNAs, lncRNAs, and circRNAs may serve as new therapeutic targets for the interaction between *E. granulosus* and the host in pathogenesis [35]. Our high-throughput sequencing data are consistent with previous results showing that miR-29c-3p and miR-30b-5p are significantly downregulated in CE [36].

Consistent with the results of previous studies, these differentially expressed molecules in infected mice are closely related to the JAK-STAT signaling pathway, PI3K-Akt signaling pathway, cell cycle, and metabolic pathways [34, 37, 38]. This implies that these pathways play an important role in promoting the growth and development of parasitism of *E. granulosus* as well as immune escape. Meanwhile, differentially expressed miRNAs, lncRNAs, and circRNAs discovered by high-throughput sequencing also affect the MAPK signaling pathway and p53 signaling pathway. MAPK signaling pathway abnormalities are thought to be closely associated with inflammatory responses [39]. In addition, the MAPK signaling pathway has a key role in the development and maintenance of parasites in the body of the host and may serve as a new therapeutic target pathway for parasitic disease [40]. Although the P53 signaling pathway is often used to study cancer-related diseases, in some parasitic infections (e.g., Plasmodium), it can reduce its parasitic burden [41, 42]. It is reasonable to assume that miRNAs, lncRNAs, and circRNAs influence *E. granulosus* infection, immune response, and pathogenesis by interacting synergistically to regulate the relevant signaling pathways and cell cycle. Further study of these interactions and pathways may provide a new perspective for the prevention and treatment of CE.

## 5. Conclusions

In this study, the use of high-throughput sequencing for RNA expression profiling of splenic CD4^+^ T cells after infection of mice with *E. granulosus* enriched our understanding of the molecular mechanisms underlying the development of CE. Although potentially important RNA molecules and associated signaling pathways were identified, further experiments and clinical trials are needed to determine their potential to serve as new targets for the treatment of CE. To obtain more meaningful and practical results, we will further verify these differentially expressed RNA molecules utilizing molecular biology techniques and explore the mechanism of their related pathways in future work. It is hoped that our work may provide a new perspective for the prevention and treatment of CE.

## Figures and Tables

**Figure 1:** (a) is the content of IFN- *γ* in the peripheral blood serum of infected and uninfected mice, (b) is the content of IL-2 in the peripheral blood serum of infected and uninfected mice, (c) is the content of IL-4 in the peripheral blood serum of infected and uninfected mice, (d) is the content of IL-6 in the peripheral blood serum of infected and uninfected mice, (e) is the content of IL-10 in the peripheral blood serum of infected and uninfected mice, (f) is the content of IL-17A in the peripheral blood serum of infected and uninfected mice, and (g) is the content of TNF-*α*in the peripheral blood serum of infected and uninfected mice.  ^*∗∗*^*P* < 0.01 (*t*-test).

**Figure 2:** Differentially expressed coding and non-coding RNAs in mouse spleen CD4^+^ T cells after *E. granulosus* infection. (a) Volcano map of differentially expressed mRNAs. (b) Cluster plots of differentially expressed mRNAs. (c) Volcano map of differentially expressed miRNAs. (d) Cluster plots of differentially expressed miRNAs. (e) Volcano map of differentially expressed lncRNAs. (f) Cluster plots of differentially expressed lncRNAs. (g) Volcano map of differentially expressed circRNAs. (h) Cluster plots of differentially expressed circRNAs. Red and green colors represent significantly upregulated and downregulated RNAs, respectively, with darker colors indicating greater degrees of alteration.

**Figure 3:** GO and pathway enrichment analyses of differentially expressed genes. GO analysis results are presented for the categories of BP, MF, and CC. (a) GO analysis of differentially expressed mRNAs. (b) Histogram of the top 15 enriched pathways of differentially expressed mRNAs. (c) GO analysis of differentially expressed circRNAs. (d) Histogram of the top 15 enriched pathways of differentially expressed circRNAs. BP, biological process; CC, cellular component; GO, Gene Ontology; MF, molecular function.

**Figure 4:** Gene act network analysis of differentially expressed genes. Red circles indicate upregulation of gene expression, green circles indicate downregulation of gene expression, and arrows indicate the direction of regulation.

**Table 1:** Top 20 significantly differentially expressed mRNA in mice with CE.

Number	mRNAs	P-value	Fold change	KEGG ID	Variation trend
1	Mogat2	≤0.001	128.593906	mmu:233549	↑
2	Slc7a2	0.004411	60.799933	mmu:11988	↑
3	Inhba	≤0.001	47.743043	mmu:16323	↑
4	Arg1	0.007749	41.718734	mmu:11846	↑
5	Svep1	0.002536	35.276715	mmu:64817	↑
6	BC100530	0.005184	25.462007	mmu:100034684	↑
7	Prok2	0.004380	24.238070	mmu:50501	↑
8	Prss57	≤0.001	22.437538	mmu:73106	↑
9	Prtn3	0.000003	21.253885	mmu:19152	↑
10	Ednrb	0.038857	18.083663	mmu:13618	↑
11	Mal	0.000243	0.004876	mmu:17153	↓
12	Morc1	0.000695	0.032526	mmu:17450	↓
13	Gm2666	0.044359	0.125757	mmu:100040213	↓
14	Phtf1	≤0.001	0.206011	mmu:18685	↓
15	Map1b	0.000004	0.190977	mmu:17755	↓
16	Il23r	0.000007	0.175867	mmu:209590	↓
17	Lhfpl3	0.000187	0.227255	mmu:269629	↓
18	Abi3bp	0.002377	0.254951	mmu:320712	↓
19	Cd46	≤0.001	0.286449	mmu:17221	↓
20	Hdgfrp3	≤0.001	0.287232	mmu:29877	↓

**Table 2:** Significantly differentially expressed miRNAs in mice with CE.

Number	miRNAs	P-value	Fold change	Variation trend
1	Mmu-miR-582-3p	≤0.001	4.801843261	↑
2	Mmu-miR-6539	0.019435	3.874091158	↑
3	Mmu-miR-6390	≤0.001	3.66410041	↑
4	Mmu-miR-223-5p	≤0.001	3.488196899	↑
5	Mmu-miR-3470a	0.000983	3.272799374	↑
6	Mmu-miR-146b-5p	0.000019	2.910612444	↑
7	Mmu-miR-340-5p	0.000908	2.654933238	↑
8	Mmu-miR-148a-3p	0.000035	2.101785735	↑
9	Mmu-miR-3470b	0.000061	2.082635327	↑
10	Mmu-miR-30a-5p	0.002306	2.046965895	↑
11	Mmu-miR-101a-3p	≤0.001	1.924605436	↑
12	Mmu-miR-152-3p	0.027217	1.905722501	↑
13	Mmu-miR-101b-3p	≤0.001	1.767716403	↑
14	Mmu-miR-7034-5p	0.013931	1.763911412	↑
15	Mmu-miR-147-3p	0.024016	1.760151814	↑
16	Mmu-miR-148a-5p	0.000004	1.721108068	↑
17	Mmu-miR-126a-3p	0.015347	1.64646616	↑
18	Mmu-miR-185-5p	0.009195	1.519753918	↑
19	Mmu-let-7f-2-3p	0.000008	0.666231102	↓
20	Mmu-miR-361-5p	0.000064	0.660195667	↓
21	Mmu-miR-30b-5p	≤0.001	0.658126995	↓
22	Mmu-miR-146a-5p	≤0.001	0.64333395	↓
23	Mmu-miR-10a-3p	0.000209	0.642253971	↓
24	Mmu-miR-27a-3p	0.000002	0.641656096	↓
25	Mmu-miR-132-3p	≤0.001	0.58349718	↓
26	Mmu-miR-191-5p	≤0.001	0.575813459	↓
27	Mmu-miR-29c-3p	0.002953	0.569357456	↓
28	Mmu-miR-30c-5p	≤0.001	0.547415662	↓
29	Mmu-miR-29a-3p	0.000006	0.539354256	↓
30	Mmu-miR-26b-3p	0.030575	0.539343428	↓
31	Mmu-miR-96-5p	0.001627	0.525567045	↓
32	Mmu-miR-664-3p	0.000001	0.48763493	↓
33	Mmu-miR-211-5p	0.004439	0.474603147	↓
34	Mmu-let-7c-2-3p	0.015834	0.469945798	↓
35	Mmu-let-7a-1-3p	0.000004	0.46446774	↓
36	Mmu-miR-455-3p	0.013980	0.401885282	↓
37	Mmu-miR-6383	0.038061	0.068552277	↓

**Table 3:** Top 20 significantly differentially expressed LncRNAs in mice with CE.

Number	LncRNAs	P-value	Fold change	Variation trend
1	Hist1h2aj	0.000001	8.365762	↑
2	BC039771	0.028185	8.151778	↑
3	Gm32462	0.025184	8.096541	↑
4	Gm36753	≤0.001	6.486906	↑
5	Cd63-ps	0.000104	5.716026	↑
6	Gm32908	0.002014	5.260593	↑
7	Terc	0.008123	4.833880	↑
8	Gm39714	≤0.001	4.769023	↑
9	Tnfsf13os	0.014627	4.214415	↑
10	Eif3s6-ps1	0.002530	0.084653	↑
11	Gm41658	0.040803	0.050741	↓
12	Gm39518	≤0.001	0.185692	↓
13	Ppp1r2-ps5	0.036916	0.145980	↓
14	LOC108169029	0.000005	0.134901	↓
15	Gm18990	0.000016	0.243135	↓
16	Gm40260	0.000199	0.214957	↓
17	Gm39807	0.000229	0.212269	↓
18	Gm15712	≤0.001	0.203890	↓
19	Hmgb1-rs16	0.005550	0.253846	↓
20	Gm40522	0.021976	0.243865	↓

**Table 4:** Significantly differentially expressed circRNAs in mice with CE.

Number	circRNAs	P-value	Fold change	Variation trend
1	Ighv1-63	≤0.001	39254.449955	↑
2	Ighv1-53	≤0.001	38661.083851	↑
3	Ighv1-64	≤0.001	33685.937287	↑
4	Ighv1-55	≤0.001	26839.405318	↑
5	Ighv1-55	≤0.001	21225.249103	↑
6	Ighv1-84	≤0.001	9951.293128	↑
7	Ighv1-33	≤0.001	9421.827989	↑
8	Spag5	0.039276	7.968195	↑
9	Ighv1-69	0.001047	5.433225	↑
10	Ighv10-3	0.000917	4.665258	↑
11	2010111I01Rik	0.000203	4.494962	↑
12	Lats1	0.032264583	4.383247	↑
13	Rev1	0.000946	4.035955	↑
14	Stat6	0.006122	3.103242	↑
15	Zcchc11	0.000314	0.319774	↓
16	Klhdc2	0.004500	0.289013	↓
17	Arhgap5	0.000073	0.229474	↓
18	Acbd5	0.000207	0.135694	↓
19	Ppp1r12a	0.000541	0.094807	↓
20	Ubn2	0.000110	0.063035	↓
21	Ighv1-55	≤0.001	0.000120	↓
22	Iglv3	≤0.001	0.000096	↓

## Data Availability

The simulation experiment data used to support the findings of this study are available from the corresponding author upon request.
